# Solving the Location Selection Problem of Self-Service Stores from the Perspectives of Sustainability and Uncertainty

**DOI:** 10.1155/2022/1518755

**Published:** 2022-09-22

**Authors:** Hao Zhang, Yuan Hou, Huixia Feng, Chenglin Xu

**Affiliations:** ^1^Beijing Technology and Business University, Beijing, China; ^2^Chinese Academy of Personnel Science, Beijing, China

## Abstract

This paper presents an improved method for selecting a specific location in the development of convenience stores in municipal areas. This method solves the problem of self-service store location from the perspective of sustainability and uncertainty and adequately considers the characteristics of individual locations with the proposition of an improved grey wolf optimization algorithm. The example presented shows that the improved algorithm has obvious advantages in facilitating the selection of convenience stores with respect to the search precision, stability, and convergence. Based on the macroenvironment, income, and cost, this work establishes a relatively complex, complete, and targeted mathematical model. Finally, taking the Xiaonanzhuang area of Suzhou Street in Beijing as an example, the scientificity, feasibility, and sustainability of the location model are verified.

## 1. Introduction

The self-service model has been studied since 2010 [1–3]. Buell et al. [4] investigated the impact of self-service technology usage on customer satisfaction and retention. Self-service terminals are used as part of a customer's checkout process in retail operations. Li et al. [5] proposed that intercustomer interactions are important for the operation of self-services in retail settings. Weretecki et al. [6] studied the impact of intercustomer interactions at retail self-service terminals on service quality perceptions and repeat purchase intentions at retail stores. Self-service stores are retail outlets in which machines replace humans in providing customers with specific services to reduce the cost of delivery and purchasing through service standardization [7, 8]. Compared with traditional retail stores, self-service stores have numerous benefits, including the use of small retail space, low inventory, the provision of convenience, and reduced operation costs [9, 10]. As a result, self-service stores have developed rapidly. The rapid development of self-service stores requires the adequate evaluation and selection of store locations in specific situations. The store location is one of the most important factors in the operation of unattended convenience stores and is directly related to their profitability. Consequently, evaluating and selecting the best store location is a critical problem that needs to be adequately addressed.

Much research has benefited from the development of specific methods for solving the site selection problem under various circumstances. Huang et al. [11] reported an analytical approach to select expansion locations for retailers selling add-on products. Moreover, the authors built predictive models for understanding the derived demand of the add-on product and established an optimization framework for automating expansion decisions to maximize expected sales. Zhao et al. [12] presented a data-driven approach to allocating ‘taxi canteens' throughout a city and proposed a constrained optimization model to select locations for these services. Mohammad and Morteza [13] presented a fast, constructive heuristic algorithm based on priority rules to determine the optimal location for storage facilities.

Rao et al. [14] proposed a fuzzy multiattribute group decision-making (FMAGDM) technique based on linguistic tuples to evaluate potential alternative CLC locations. Birol [15] proposed the Fuzzy Preference Ranking Organization method for enrichment evaluation to evaluate the potential location of logistics centers. Such methods in general can be classified as multiple criteria decision-making (MCDM) methods, mathematical methods, and intelligent methods. MCDM methods always involve multiple objectives, there are contradictions and incommensurability among objectives, and the qualitative and quantitative indicators are mixed [16–18]. The multicriteria decision siting model often contains some specific constraints, can satisfy multiple objectives, and focuses on comprehensively considering multiple criteria for nuclear site selection [19]. Rouyendegh and Savalan [20] combine multiple-criteria decision-making with an analytic hierarchy process and fuzzy sets to establish a hybrid model to provide decision support for the selection of sustainable solutions to agricultural problems. Ghosh et al. [21] studied the application of the hexagonal fuzzy multicriteria decision-making method in the location of charging stations for electric vehicles. Erol et al. [22] proposed a new decision-making framework based on fuzzy MCDM to sort the site selection of alternative nuclear power plants in Turkey. As a result of the existence of qualitative indicators, this method is greatly influenced by subjective factors. In actual decision-making, these qualitative indicators must be treated with fuzzy quantification.

Mathematical methods are used to solve location selection problems by quantifying factors such as costs and expenses, defining definite assumptions, setting parameters and variables, and establishing a mathematical model for optimization [23, 24]. The entropy weight method and TOPSIS model are used to determine distribution center locations in cold-chain logistics. From the perspective of quantitative analysis, how comprehensive factors influence the site selection problem is difficult to consider by establishing a mathematical model for solving it, such as topography, land appreciation, urban development, environment, traffic, pollution, and the impact on the user, which usually cannot be quantified and ignored. The use of mathematical methods to solve practical problems with large amounts of data is often difficult. Mathematical models are always ideal and precise.

The emergence of intelligent algorithms has greatly enriched modern optimization technology and provided practical solutions for combinatorial optimization problems that are difficult to solve using traditional optimization techniques, such as genetic algorithms, particle swarm algorithms, and differential evolution algorithms [25, 26]. These methods share many of the same characteristics: (1) all indeterminate algorithms; (2) global optimization algorithms; (3) excellent distributed computing mechanisms; (4) self-organization and evolution; and (5) strong robustness; however, some defects exist, such as (1) the accuracy of the solution results is often sacrificed for the efficiency of the solution; (2) it easily falls into the local optimal solution; and (3) the selection of algorithm parameters is based mainly on experience.

As a new type of offline retail business, there are few research papers on unmanned convenience stores, and few researchers participate in the study of the operation and management of unmanned convenience stores. At present, the existing research articles on unmanned convenience store mainly focus on analyzing its market positioning and its own operating characteristics and summarize the current development of the industry. Based on this, a self-service store location model is proposed, and an improved grey wolf optimization (GWO) algorithm is proposed to solve the model. Aiming at the improvement strategy of global optimization algorithm, an endogenous improvement method is proposed to optimize the application of global optimization algorithm in linear programming computational problems. The factors affecting the location of self-service stores are analyzed. Seven representative influencing factors are proposed, and two hypotheses are put forward: store rent is the revenue factor, and daily flow is the cost factor. Horizontal competitors in the surrounding area assist in the operation of self-service stores. These hypotheses are verified by practical cases, and their rationality and practical significance are demonstrated.

The remainder of the paper is divided into four sections. The next section describes the location problem and the associated factors. The improved grey wolf algorithm is introduced to solve the mathematical model of the location problem and runs tests using the class functions. A location model of convenience stores is established against this improved algorithm backdrop. This step is followed by selecting the location of two convenience stores in Beijing, and the results of the location model are analyzed. Finally, the concluding section details some practical suggestions for improving future site planning.

## 2. Formulating the Selection Problem

After analyzing many references and conducting field research in Beijing, the following factors influencing the location selection of self-service stores were summarized to establish the location selection model:

### 2.1. Environmental Factors

Environmental factors should include the specific location of the reserved location, specific area, degree of policy support, degree of macroregional development, and degree of development of social law and morality [27]. These factors are generally predetermined.

### 2.2. Revenue Factor

The revenue factor is an important factor that can, directly and indirectly, influence the operating profit of self-service stores. Profit is how much revenue exceeds the cost [28]. The profit of the enterprise comes directly from consumers' consumption in the store.

### 2.3. Cost Factors

The cost factors generally include the site cost, goods loss cost, maintenance and replacement cost, depreciation cost, and manpower cost [29, 30]. The model of this paper should include the daily flow of people, distance from dangerous areas, maintenance distance, and several peripheral competitors. Self-service stores prefer small numbers of customers with high net worth and long-term stable demand. Therefore, too much traffic does not have a positive effect on these stores. In contrast, due to its limited space, limited reception capacity, and the consumption of hardware facilities and products, too much traffic will have a highly negative impact. Therefore, the people flow is a cost factor with a large changed weight.

Location in a potentially dangerous area is a serious cost factor. Such an area can attract people who do not intend to shop at the convenience store, create discomfort, and feature low-quality facilities and the potential harm to the store or customers. This factor should therefore be heavily weighted. Surrounding competitors represent the competition factor. Peripheral competitors will inevitably affect the store's income level, but there are no convenience stores with general offline retail stores. Sales are not repelled but increased around a certain number of traditional offline retail stores, as the presence of competitors increases the main demand of passenger flow and disperses them; therefore, this cost factor has a smaller weight. Maintenance distance is the distance from the warehouse to the location of the staff responsible for maintaining the self-service store. The space affects warehouse sales and self-service stores and is affected by the total number of warehouses. Then, the model should consider all preexisting warehouses and no convenience store randomness. The characteristics of the high-frequency replenishment and exchange of goods mean that the distance should be as low as possible. Thus, this factor is a cost factor.

### 2.4. Correlation Factors

Correlation factors refer to the interactions between factors. The main correlation factors are as follows;

#### 2.4.1. Associated Effects of the Master Stream Band

When the site location is closer to the mainstream of people, away from residential and office areas, the income-weighted rent cost for peripheral small village land is low, and the weight of the cost factor of daytime traffic is large. Conversely, when the location is away from the mainstream of people and close to residential and office areas, the income-weighted rent cost for peripheral districts is larger, with a smaller value for the weight of the cost factor of daytime traffic.

#### 2.4.2. Associated Effects of Risky Areas

When a location is too close to a dangerous area, the weight of daytime human flow and the distance to the dangerous area will correspondingly increase. In contrast, when the location's proximity to a dangerous area meets the specified limit, the weight of the daytime human flow and the distance to the dangerous area will correspondingly decrease.

#### 2.4.3. Associated Effects of Distance to the Maintenance Area

When the location is too far from the maintenance area, the weight of the daytime human flow and distance to the maintenance area will correspondingly increase. In contrast, when the location's distance to a dangerous area meets the specified limit, the weight of daytime human flow and distance to the maintenance area will decrease.

## 3. Formulating the Site Selection Problem

The objective function of the optimal location is expressed as follows:

(1) $$\begin{array}{c} P_{\text{best}}=\text{MAX}\left(P_{i}\right), \end{array}$$

where P_*i*_ is the optimal location searched by the algorithm in each iteration, which can be expressed as

(2) $$\begin{array}{c} P_{i}=\text{L}{\text{P}}_{i}+R_{i}+\text{D}{\text{F}}_{i}+\text{N}{\text{F}}_{i}+\text{D}{\text{Z}}_{i}+\text{C}{\text{N}}_{i}+\text{M}{\text{D}}_{i}+Z_{i}, \end{array}$$

where LP_*i*_, *R*_*i*_, DF_*i*_, NF_*i*_, DZ_*i*_, CN_*i*_, MD_*i*_, and *Z*_*i*_ are represented as different total weight values at position *i*, which are detailed as follows:

1. LP_*i*_ is the total weight value of the land price in the neighbourhood of the community at position *i*, which should be expressed as

(3) $$\begin{array}{c} \text{L}{\text{P}}_{i}=\text{L}{\text{P}}_{w}\times \text{L}{\text{P}}_{c_{i}}\times \text{LP}{\text{K}}_{i}\times \text{DP}{\text{a}}_{i}, \end{array}$$

where LP_*w*_ is the default weight of the land price, LPc_*i*_ is the normalized value of the practical land price at position *i*, and LPk_*i*_ is the dependency coefficient of the actual location on the land price, which can be expressed as

(4) $$\begin{array}{c} \text{LP}{\text{K}}_{i}=\left\{\begin{array}{c} \omega_{1}\\ \theta_{1} \end{array}\right.\;\begin{array}{c} \text{dd}\leq \text{DD},\\ \text{dd}>\text{DD}, \end{array}\\ \text{DP}{\text{a}}_{i}=\left\{\begin{array}{c} \alpha_{1}\\ \beta_{1} \end{array}\right.\;\begin{array}{c} \text{p}{\text{p}}_{i}\subset \text{DP},\\ \text{p}{\text{p}}_{i}⊄\text{DP}, \end{array} \end{array}$$

where *ω*_1_ and *θ*_1_ are different constants. dd is the distance from the location to the nearest master stream belt, and DD is the default distance limit. DPa_*i*_ is the influence coefficient of the closed area on the surrounding land price, while *α*_1_ and *β*_1_  are different constants, pp_*i*_ is the location of the prelocation, and DP is the closed area.

(2) R_*i*_ is the total weighted value of the store's rent in location *i*, which can be expressed as

(5) $$\begin{array}{c} R_{i}=R_{w}\times {\text{Rc}}_{i}\times \text{R}{\text{k}}_{i}, \end{array}$$

where *R*_*w*_ is the default weight of the store's rent, Rc_*i*_ is the normalized value of the actual rent, and Rk_*i*_ is the dependency coefficient of the actual location on the rent, which can be represented as

(6) $$\begin{array}{c} \text{R}{\text{K}}_{i}=\left\{\begin{array}{c} \omega_{2}\\ \theta_{2} \end{array}\right.\;\begin{array}{c} \text{dd}\leq \text{DD},\\ \text{dd}>\text{DD}, \end{array}\\ \text{DP}{\text{b}}_{i}=\left\{\begin{array}{c} \alpha_{2}\\ \beta_{2} \end{array}\right.\;\begin{array}{c} \text{p}{\text{p}}_{i}\subset \text{DP},\\ \text{p}{\text{p}}_{i}⊄\text{DP}, \end{array} \end{array}$$

where *ω*_2_ and *θ*_2_ are different constants. DPb_*i*_ is the influence coefficient of the closed area on the surrounding land price, while *α*_2_ and *β*_2_  are different constants.

(3) DF_*i*_ is the total weighted value of the daytime flow of people at position *i*, which can be expressed as

(7) $$\begin{array}{c} \text{D}{\text{F}}_{i}=\text{D}{\text{F}}_{w}\times \text{DF}{\text{c}}_{i}\times \text{DF}{\text{k}}_{i}\times \text{C}{\text{O}}_{i}, \end{array}$$

where DF_*w*_ is the fixed weight of the daytime flow, DFc_*i*_ is the normalized value of actual daytime flow at position *i*, DFk_*i*_ is the dependence coefficient of the actual location on the flow of people at position *i*, and CO_*i*_ is the influence coefficient of the number of competitors on the daytime flow, which can be described as

(8) $$\begin{array}{c} \text{DF}{\text{K}}_{i}=\left\{\begin{array}{c} \omega_{3}\\ \theta_{3} \end{array}\right.\;\begin{array}{c} \text{dd}\leq \text{DD},\\ \text{dd}>\text{DD}, \end{array}\\ \text{C}{\text{O}}_{i}=\left\{\begin{array}{cc} 1 & \sum \text{c}{\text{n}}_{ic}=0,\\ \mu_{1} & \sum \text{c}{\text{n}}_{ic}=1,\\ \mu_{2} & \sum \text{c}{\text{n}}_{ic}=2, \end{array}\right.\\ \text{c}{\text{n}}_{ic}=\left\{\begin{array}{c} 1\\ 0 \end{array}\right.\;\begin{array}{c} \text{dc}{\text{c}}_{i}\leq \text{dcd},\\ \text{dc}{\text{c}}_{i}>\text{dcd}, \end{array}\\ \text{DP}{\text{c}}_{i}=\left\{\begin{array}{c} \alpha_{3}\\ \beta_{3} \end{array}\right.\;\begin{array}{c} \text{p}{\text{p}}_{i}\subset \text{DP},\\ \text{p}{\text{p}}_{i}⊄\text{DP}, \end{array} \end{array}$$

where *ω*_3_ and *θ*_3_ represent different constants. CO_*i*_ is the influence coefficient of the number of competitors on the daytime flow. 1 < *μ*_1_ < *μ*_2_, and they are all constants. cn_*ic*_ is the number of competitors in the default distance dcc_*i*_ of position *i*. DPc_*i*_ is the influence coefficient of the closed area on the daytime flow, and *α*_3_ and *β*_3_ are different constants.

(4) NF_*i*_ is the total weighted value of the night flows at position *i*, which should be expressed as

(9) $$\begin{array}{c} \text{N}{\text{F}}_{i}=\text{N}{\text{F}}_{w}\times \text{N}{\text{Fc}}_{i}, \end{array}$$

where NF_*w*_ is the default weight of the flow of people at night, and NFc_*i*_ is the normalized value of the actual night flow at position *i*. Because the stream of people at night is relatively lower than that during the day and the service objects are mostly local residents, the cost of loss is lower. In this context, because of the sudden demand of customers and the irreplaceability of self-service stores for general stores, the store earnings rise as the number of customers increases.

(5) DZ_*i*_ is the total weighted value of dangerous areas at position *i*, which can be expressed as

(10) $$\begin{array}{c} \text{D}{\text{Z}}_{i}=\text{Rw}\times \text{R}{\text{c}}_{i}\times \text{DZ}{\text{k}}_{i}, \end{array}$$

where Rw is the default weight of the store's rent, Rc_*i*_  is the normalized value of the actual rent, and DZk_*i*_ is the dependency coefficient of the actual location on the dangerous area, which can be represented as

(11) $$\begin{array}{c} \text{DZ}{\text{K}}_{i}=\left\{\begin{array}{cc} \omega_{4} & \text{dd}{\text{z}}_{i}\leq \text{DDZ},\\ \theta_{4} & \text{dd}{\text{z}}_{i}>\text{DDZ}, \end{array}\right. \end{array}$$

where *ω*_4_ and *θ*_4_ represent different constants. dd*z*_*i*_  is the distance between location *i* and the nearest dangerous area, and DDZ is the default distance limit.

(6) CN_*i*_ is the total weighted value of regional competitors in position *i*, which can be expressed as

(12) $$\begin{array}{c} \text{C}{\text{N}}_{i}=\text{C}{\text{N}}_{w}\times \text{C}{\text{Nc}}_{i}, \end{array}$$

where CN_*w*_ is the default regional competitor weight and CNc_*i*_ is the normalized value of the actual number of regional competitors in position *i*.

(7) MD_*i*_ is the total weighted value of the maintenance distance at location *i*, which can be expressed as

(13) $$\begin{array}{c} \text{M}{\text{D}}_{i}=\text{M}{\text{D}}_{w}\times \text{M}{\text{Dc}}_{i}\times \text{MD}{\text{k}}_{i}, \end{array}$$

where  MD_*w*_ is the weight of the default maintenance distance and MDc_*i*_ is the normalized value of the actual maintenance distance at position *i*. MDk_*i*_ is the dependence coefficient of the actual location on the distance to the maintenance area, which can be represented as

(14) $$\begin{array}{c} \text{MD}{\text{K}}_{i}=\left\{\begin{array}{c} \omega_{5}\\ \theta_{5} \end{array}\right.\;\begin{array}{c} {\text{ddm}}_{i}\leq \text{DDM},\\ {\text{ddm}}_{i}>\text{DDM}, \end{array} \end{array}$$

where *ω*_5_ and *θ*_5_ represent different constants. ddm_*i*_  is the distance between location *i* and the nearest dangerous area, and DDM is the default distance limit.

## 4. A New Method

Grey wolves are highly intelligent social animals and have long been considered a dangerous top predator, which means they are at the top of the food chain. Most grey wolves like to live in a small cluster.

The leader of the herd can be a male wolf or a female wolf, which we call the alpha (*α*) wolf. Alpha (*α*) wolves are mainly responsible for making decisions about where the population hunts, where they sleep, when they wake up, and so on. The decision of the alpha (*α*) wolf depends on individual thinking and decision-making behaviour [31]. However, biologists have also observed some kind of democratic behaviour; that is, alpha (*α*) wolves sometimes follow other subordinate wolves. In the group, the whole population recognizes the alpha (*α*) by raising its tail. The alpha (*α*) wolf is also called the dominant wolf because his or her orders should be obeyed by the whole pack. Alpha (*α*) wolves are only allowed to mate and reproduce in their own population. It is worth noting that alpha (*α*) wolves are not necessarily the strongest and most ferocious members of the pack, but they are the best at managing the pack [32]. This shows that for the first wolf, that is, alpha (*α*) wolf, organizational ability and discipline are much more important than their individual strength in status evaluation.

The second level of the grey wolf class is the beta (*β*) wolf. Beta (*β*) wolves are subordinate wolves to help alpha (*α*) wolves make decisions or leaders of other ethnic activities. Beta (*β*) wolves can be either male or female, and he or she may be the best candidate for alpha (*α*) wolves to prevent the death or aging of alpha wolves. Beta (*β*) wolves should respect the alpha (*α*), but also command and command other lower-level wolves. It plays the role of consultant and trainer. Beta (*β*) wolves play a role in strengthening the alpha (*α*) command and providing feedback to the alpha (*α*) in the whole population [33, 34].

The lowest ranking grey wolf is the omega (*ω*) wolf. Omega (*ω*) plays the most passive role of scapegoat. Omega wolves always have to obey all other higher-level dominant wolves. They are the last wolves allowed to hunt and feed. Omega (*ω*) wolves may not seem like a very important hierarchy, but biologists have observed the problems caused by internal fighting and the loss of omega (*ω*) wolves in the entire population [35]. This is because omega (*ω*) wolves mainly perform the function of violence and destruction at all levels of the pack. This helps to meet the needs of the whole ethnic group and maintain the dominant structure. In some cases, omega (*ω*) is also a maintainer in the community.

If the selected grey wolf is not an alpha (*α*) wolf, a beta (*β*) wolf, or an omega (*ω*) wolf, then he or she is called a delta (*δ*) wolf. Delta (*δ*) wolves must obey the alpha (*α*) wolves and the beta (*β*) wolves, but they will dominate the omega (*ω*) wolves. Scouts, sentinels, elders, hunters, and guards belong to the role of this type of wolf. The scouts are responsible for monitoring the boundaries of the territory and warning the guard in the event of danger. The sentry protects and ensures the safety of the packing [36]. Elders are experienced wolves who used to be alpha (*α*) wolves or beta (*β*) wolves. Hunters help the alpha (*α*) wolves and the beta (*β*) wolves when hunting prey and providing food. Finally, the guards are responsible for taking care of the weak, sick, and injured members of the pack. In the GWO algorithm, the hunter-gatherer (optimization) is always led by *α*, *β*, and *δ*. The rest of the wolves follow these three wolves. According to the description of Muro et al. [37] the main stages of grey wolf hunting are as follows:

1. Tracking, chasing, and approaching prey
2. Pursuing, surrounding, and harassing the prey until it stops moving
3. Attacking the prey

Grey wolves surround their prey during hunting. To simulate surrounding behaviour mathematically, the following equation is proposed:

(15) $$\begin{array}{c} \overset{⟶}{D}=\left|\overset{⟶}{C}\times \overset{⟶}{X_{p}}\left(t\right)-\overset{⟶}{X}\left(t\right)\right|,\\ \overset{⟶}{X}\left(t+1\right)=\overset{⟶}{X_{p}}\left(t\right)-\overset{⟶}{A}-\overset{⟶}{D,} \end{array}$$

where *t* represents the current iteration, $\overset{⟶}{A}$ and $\overset{⟶}{C}$ are coefficient vectors, ${\overset{⟶}{X}}_{p}\left(t\right)$ is the position vector of prey, and $\overset{⟶}{X}$ indicates the position vector of grey wolves.

(16) $$\begin{array}{c} \overset{⟶}{A}=2\overset{⟶}{a}\times \overset{⟶}{r_{1}}-\overset{⟶}{a}, \end{array}$$

(17) $$\begin{array}{c} \overset{⟶}{C}=2\overset{⟶}{r_{2}.} \end{array}$$

In the iterative process, the convergence factor decreases linearly from 2 to 0, and the vector *r* is the random number between 0 and 1. Grey wolves can update the position in the surrounding space of their prey at any random position using equations (16) and (17).

We save the first three best solutions so far and ask the other search agents (including the omega wolf) to update their location *X*_*α*_, *X*_*β*_, and *X*_*δ*_ according to the position of the optimal search agent:

(18) $$\begin{array}{c} \begin{array}{c} x_{i,\alpha }^{d}\left(t+1\right)=X_{\alpha }^{d}\left(t\right)-A_{i,1}^{d}\left|C_{i,1}^{d}X_{\alpha }^{d}\left(t\right)-X_{i}^{d}\left(t\right)\right|,\\ x_{i,\beta }^{d}\left(t+1\right)=X_{\beta }^{d}\left(t\right)-A_{i,2}^{d}\left|C_{i,2}^{d}X_{\beta }^{d}\left(t\right)-X_{i}^{d}\left(t\right)\right|,\\ x_{i,\delta }^{d}\left(t+1\right)=X_{\alpha \delta }^{d}\left(t\right)-A_{i,3}^{d}\left|C_{i,3}^{d}X_{\alpha \delta }^{d}\left(t\right)-X_{i}^{d}\left(t\right)\right|, \end{array}\\ X_{i}^{d}\left(t+1\right)=\frac{X_{i,a}^{d}\left(\text{t}+1\right)+X_{i,\beta }^{d}\left(t+1\right)+X_{i,\delta }^{d}\left(t+1\right)}{3}, \end{array}$$

where *X*_*i*_^*d*^(*t* + 1) represents the fitness value of the individual grey wolf *i* in generation *t* + 1.

To solve the problem that the basic GWO easily falls into a local optimum, this paper improves two aspects:

### 4.1. Convergence Factor Strategy Based on Nonlinear Decline

In GWO, the default convergence factor decreases linearly from 2 to 0 as the number of iterations increases; however, in using the actual algorithm and solving the function, the algorithm convergence trend is not linear. Therefore, the linear decreasing strategy of convergent factor in the basic algorithm is not completely suitable for the actual algorithm when searching and calculating the optimal value of the function. Therefore, a new nonlinear convergence method is proposed in this paper:

(19) $$\begin{array}{c} a=2-2{\left(\frac{l}{n}\right)}^{2}, \end{array}$$

where *l* is the current iteration number; *n* is the default maximum number of iterations; and *a* is a nonlinear convergence factor.

The nonlinear convergence of convergence factor *a* is shown in figure 1.

When the maximum number of iterations is 500, the blue function curve represents the speed of basic GWO convergence, and the red function curve represents the speed of optimized algorithm convergence. The improved convergence factor *a* presents the curve convergence with the iterations; in the short term, a slow convergence speed can interact with the GWO to determine a better global optimal solution, and in the medium term, the convergence of the algorithm is accelerated. The convergence speed of *a* accelerates at the later stage, which helps the algorithm find the local optimal solution quickly.

### 4.2. Fixed Penalty Function Method for Multisegment Association Mapping

Because GWO is an optimization algorithm search technology based on an unconstrained function, it is necessary to combine an appropriate constraint treatment when solving the optimization problem of the constrained function with GWO. The penalty function method is most commonly used to handle a series of unconstrained optimization algorithm technologies.

As shown in equation (20), the constraint optimization problem is as follows:

(20) $$\begin{array}{c} \begin{array}{c} \text{Min}f\left(x\right),\\ \text{s}.\text{t}.g_{j}\left(x\right)\leq 0\;j=1,2,3,\cdots ,p,\\ h_{j}\left(x\right)=0\;j=p+1,p+2,p+3,\cdots ,m,\\ l_{i}\leq x_{i}\leq u_{i}\;i=1,2,3,\cdots ,d, \end{array} \end{array}$$

where *f*(*x*) is the target function,  *g*_*j*_(*x*) is the constraint condition of the inequality, *h*_*j*_ (*x*) is the constraint condition of the equation, and *l*_*i*_ and *u*_*i*_ are the upper and lower bounds of the variable *x*_*i*_, respectively.

This equation can be translated into the following form:

(21) $$\begin{array}{c} \begin{array}{c} h_{j}\left(x\right)-\varepsilon \leq 0,\\ -h_{j}\left(x\right)-\varepsilon \leq 0, \end{array} \end{array}$$

where *ε* is called the tolerance value, which is generally taken as a small positive number. The general form of the constructed generalized objective function is as follows:

(22) $$\begin{array}{c} F\left(x\right)=f\left(x\right)+\partial \left(t\right)H\left(x\right), \end{array}$$

where *F*(*x*) is the original target function, partial *∂*(*t*)*H*(*x*) is called the punishment term, partial *∂*(*t*) is expressed as the punishment intensity, and *H*(*x*) is called the punishment factor.

During the whole process of solving the optimization problem of constraints, if the partial (*t*) in equation (22) is fixed, it is called the fixed penalty function method; otherwise, it is called the nonfixed penalty function method. The fixed penalty function method will be determined by a set of preset parameters in accordance with the actual situation or theoretical situation and will not change due to changes in the number of iterations. Multisegment mapping is when the function value or variable value changes, and the default constraint function will have different constraint effects on the original function, which is expressed as:

(23) $$\begin{array}{c} \begin{array}{cc} H_{1}\left(x\right)=A\left(x\right)\times B\left(x\right), & \\ A_{1} & A\left(x\right)\leq r_{1},\\ A_{2} & r_{1}<A\left(x\right)\leq r_{2},\\ A_{3} & r_{2}<A\left(x\right)\leq r_{3,} \end{array} \end{array}$$

where *H*_1_(*x*) is the target punishment function; *A*(*x*) is the punishment intensity; *B*(*x*) is the punishment degree; *A*_1_, *A*_2_, and *A*_3_ are the punishment intensity set; and *r*_1_, *r*_2_, and *r*_3_ are the upper and lower bounds of different sections.

The correlational penalty function can be expressed as

(24) $$\begin{array}{c} \begin{array}{c} H_{2}\left(x\right)=A_{2}\left(x\right)\times B_{2}\left(x\right),\\ H_{3}\left(x\right)=A_{3}\left(x\right)\times B_{3}\left(x\right), \end{array}\\ \begin{array}{cc} \text{A}{\text{X}}_{2} & x<e_{1},\\ \text{B}{\text{X}}_{2} & x\geq e_{1},\\ \text{A}{\text{X}}_{3} & H_{2}\left(x\right)<e_{2},\\ \text{B}{\text{X}}_{3} & H_{2}\geq e_{2}, \end{array} \end{array}$$

where *H*_2_(*x*) and *H*_3_(*x*) are objective functions; *A*_2_(*x*) and *A*_3_(*x*) are weights of punishment; *B*_2_(*x*), *B*_3_(*x*), and *r* are the reference boundary of the independent variable *x*; AX_2_ and BX_2_ are variable values of presupposed *A*_2_(*x*); and *e*_2_ is the reference boundary of the dependent variable*H*_2_(*x*). AX_3_ and BX_3_ are the variable presupposed values of dependent variable *H*_2_(*x*).

According to the above ideas and formulas, a new grey wolf optimization algorithm is proposed in this paper, and its process can be summarized as follows. The flow chart is shown in Figure 2.

**Step 1 .**

Initialize the grey wolf population, that is, randomly generate the position of *n* intelligent individuals; initialize *a*, *A*, and *C*; initialize the value of *X*_*α*_, *X*_*β*_, and *X*_*δ*_.

**Step 2 .**

The transboundary intelligent individual is processed, and the fitness value of each intelligent individual is calculated.

**Step 3 .**

Compare the fitness of each individual of intelligence, and determine the optimal solution, optimal solution, suboptimal solution, and *X*_*α*_, *X*_*β*_, and *X*_*δ*_in the current iteration.

**Step 4 .**

For each intelligent individual, the strategy is adjusted nonlinearly according to the control parameters, and the parameters *a* are obtained by optimization, and then *A* and *C* are obtained.

**Step 5 .**

According to the optimized position determination method and the nonlinear penalty function, the position of the intelligent individual is redetermined.

**Step 6 .**

Then, determine the fitness of the new generation of individuals and update the population level.

**Step 7 .**

If the end condition (maximum number of iterations) is reached, the end is finished and the optimal solution is output, otherwise go to Step 2.

## 5. Simulation Study

To test the feasibility and practical reliability of the IGWO, we used classic test functions, including unimodal functions and multipeak functions. Each function was used to extract three sample tests and was compared with GWO and PSO. The details are shown in Tables 1 and 2:

Each test function was tested at least 50 times, and the representative image was taken for display. The details are shown in Figures 3–8.

As shown, compared to PSO, IGWO has obvious advantages in terms of speed and precision and does not easily fall into the local optimum. IGWO shows clear superiority of the functional testing results shown in Table 3.

Table 3 shows the following aspects in detail:

### 5.1. Evaluation of exploitation capability (functions F_1_–F_3_)

Functions F_1_–F_3_ are unimodal with only one global optimum, which can evaluate the exploitation capability of the investigated metaheuristic algorithms. According to the results in the table, the present algorithm provides very good exploitation.

### 5.2. Evaluation of exploration capability (functions F_4_–F_6_)

To evaluate the exploration capability of an optimization algorithm, we used multimodal functions. These functions include many local optima whose number increases exponentially with the problem size (the number of design variables).

In terms of quantitative analysis, on the premise of keeping the original search time unchanged, the improved grey wolf optimization algorithm improves the search accuracy by 100%. The search accuracy of all test functions of PSO, PSO, and GWO can only be maintained to about *e*^−28^, while the improved grey wolf optimization algorithm can stably improve the search accuracy to about the maximum *e*^−60^, and performs well in several test functions, significantly leading the accuracy of GWO and PSO. In fact, because the algorithm slows down the convergence speed of the convergence factor in the early stage, the algorithm actually searches more possible solutions and traverses more possibility intervals, so the actual operation speed of the algorithm is accelerated. It shows its extremely high precision and not easy to fall into the local optimal performance.

In terms of qualitative analysis, the improved grey wolf optimization algorithm further improves the convergence speed and the smooth degree of convergence in the second half of the algorithm on the premise of keeping the original convergence curve from deterioration. IGWO further maintains and improves its own characteristics of fast iteration speed, fast convergence speed, and fast search speed in the process of comparing PSO and GWO.

## 6. Examples

### 6.1. Case Analysis

The case area is zoned from the auxiliary road of Wanquanhe Road in the north to Suzhou Street in the south and from western Sanyimiao Community in the east to Wanliu East Road in the west. The area is 1.2 km long from east to west, the longest distance from north to south is 900 m, and the shortest is 650 m. The case area contains a total of eight residential areas, including Guangda Garden, Xiaonanzhuang Community, and Xinjiyuan Space, two primary schools, two secondary schools, and a floating population area. An illustration of the area is shown as Figure 9.

To build the model, the area was transformed into a rectangle with a length of 120 and a width of 80, and each optional location in the region was marked. The dangerous area is marked in blue, the maintenance area is marked in green, and surrounding competitors are marked in red. The approximation is as follows Figure 10.

Through the measurement of the actual model described in the previous chapter, we obtained seven kinds of data for seven areas, as shown in Table 4, then, we normalized the data.

We then introduced a linear normalization formula to normalize the data used in this paper:

(25) $$\begin{array}{c} P_{i}^{*}=\frac{P_{i}-P_{\max}}{P_{\min}-P_{\max}}, \end{array}$$

(26) $$\begin{array}{c} P_{i}^{*}=\frac{P_{i}-P_{\min}}{P_{\max}-P_{\min}}, \end{array}$$

where *P*_*i*_ is the *i*-th value of the *P* class data. *P*_max_ refers to the maximum value of the *P* class data, *P*_min_ refers to the minimum value of the *P* class data, and *P*_*i*_^∗^ is the normalized value of the *i*-th value of the *P* class data. Formula (25) is used when *P*_*i*_ is smaller and closer to the expected situation. Formula (26) is used when *P*_*i*_ is larger and closer to the expected situation.

In practical application, taking area 1 (Xiaomai) as an example when calculating the land price factor, this factor increases as it becomes closer to the expected value, which can be written as

(27) $$\begin{array}{c} A_{1}^{*}=\frac{4.6-5.5}{4.3-5.5}=0.25, \end{array}$$

However, when normalizing the value of the distance from the danger area, this factor decreases as it becomes closer to the expected value, which can be written as

(28) $$\begin{array}{c} E_{1}^{*}=\frac{5-5}{1-5}=0. \end{array}$$

This process is similar to the remaining data.

### 6.2. Analysis of the Model Calculation Results

MATLAB software was used for 200 tests (as in the previous procedure) to form the scatter diagram of location selection shown in Figure 11; that is, the optimal solution to the location selection problem. The optimal locations are mainly concentrated in the Youth Apartment area (enclosed residential area) in area 4 and the office building in area 5. In these areas, the floating population is low, which guarantees that the customer source is active and stable; however, the land price of the neighborhood around area 7 is high, as the area features mainly residents with higher incomes. The area is close to the planned maintenance location for urban and rural storage, which helps to reduce maintenance costs. Conforming with the self-service retail industry in Beijing before the existing location mode emphasizes the main principles to “avoid crowds, implement closed-end management, serve select customer groups, implement low flow operations, and be close to maintenance areas;” this approach can ensure the long-term stable development of self-service stores.

## 7. Conclusion

In this paper, IGWO is proposed. This approach features high stability, high speed, accuracy, and global scope, can solve the optimal search problem of the related functions involved in the general swarm intelligence optimization algorithm, and has good adaptability and reliability for common functions. This paper also tries to solve the problem of convenience store location from the perspective of sustainability and uncertainty, and explores the development history of the unmanned retail industry in China, focuses on the development process of the self-service store industry in Beijing, and analyses the development of several typical self-service stores in Beijing and the location of these sites.

Based on research and analysis, three categories of dimensions are summarized:

1. Macroenvironmental factors, which include policy factors, legal and quality factors, macroeconomic development factors, and the specific circumstances of the selected regions
2. Income factors, which include land price, shop rent, and night flow
3. Cost factors, which include daytime flow, risk zone distance, maintenance area distance, and surrounding competitors

Through these dimensions, a relatively complex, sustainable, complete, and targeted mathematical model has been established. Finally, we selected Suzhou Street in the Xiaonanzhuang area as a case area and verified the scientific feasibility of the location model.

### 7.1. Managerial Insights

The problem of determining the location of convenience stores has often been mentioned by previous researchers but without a scientific, systematic, visual, and quantifiable description or calculation method to address it. In response, an effective, targeted, systematic, and practical location method is proposed in this paper. In terms of optimization and improvement strategies for the grey wolf optimization algorithm, some endogenous improvement methods are provided, and the calculation of the linear programming problem is optimized. These advancements offer innovation, pertinence, and practicability. For the establishment of the location model for convenience stores, seven representative important influencing factors are put forward, and two hypotheses are proposed: store rent is a factor of income, and the flow of people in the daytime is a factor of cost, and competitors in the surrounding industry are helpful for the operation of the convenience store. Using an actual case to verify these assumptions, we proved their rationality and practical significance.

### 7.2. Opportunities for Future Research

This paper focuses on improving the internal mechanism of the GWO algorithm. The algorithm's optimization speed is not optimal and thus room for improvement remains to avoid falling into local optimization. At present, the most popular method is to use two or more hybrid algorithms, such as hybrid difference algorithms and genetic algorithms, to improve this optimization. Future research can integrate multiple algorithms to overcome the problem of easily falling into local optimization.

For convenience, this paper focuses mainly on factors that can be simply quantified and have fixed values. For some content, it is difficult to investigate and collect information, including the impact of the population age ratio on consumption in the convenience store, the consumption tendency of customers at the convenience store, and the subjective attraction of the location to the crowd. These factors have not been investigated, analyzed, and evaluated in depth, which makes the evaluation ability of the mathematical model in the subjective direction insufficient. Future researchers can conduct more in-depth analyses of these aspects.

## Figures and Tables

**Figure 1:** Comparison of convergence factors.

**Figure 2:** Flow chart of improved grey wolf optimization algorithm.

**Figure 3:** *f*_1_ = ∑_*i*=1_^*n*^*x*_*i*_^2^ test function.

**Figure 4:** *f*_2_ = ∑_*i*=1_^*n*^|*x*_*i*_| + ∏_*i*=1_^*n*^|*x*_*i*_| test function.

**Figure 5:** *f*_3_ = ∑_*i*=1_^*n*^(∑_*j*−1_^*i*^*x*_*j*_)^2^ test function.

**Figure 6:** *f*_4_ = ∑_*i*=1_^*n*^[*x*_*i*_^2^ − 10cos(2*πx*_*i*_)] + 10 test function.

**Figure 7:** $f_{5}=-20\exp\left(-0.2\sqrt{\left(1/n\right)\sum_{i=1}^{n}x_{i}^{2}}\right)-\exp\left(\left(1/n\right)\sum_{i=1}^{n}\cos\left(2\pi x_{i}\right)\right)+20+e$ test function.

**Figure 8:** $f_{6}=\left(1/4000\right)\sum_{i=1}^{n}x_{i}^{2}-\prod_{i=1}^{n}\cos\left(x_{i}/\sqrt{i}\right)+1$ test function.

**Figure 9:** Location map for Xiaomai (Suzhou Street).

**Figure 10:** Segmentation of the Xiaomai site selection area.

**Figure 11:** Site selection result for Xiaomai (Suzhou Street).

**Table 1:** Unimodal function.

Function	Dim	Range	*f*_min_
$f_{1}=\overset{n}{\underset{i=1}{\sum }}x_{i}^{2}$	30	[-100,100]	0
$f_{2}=\overset{n}{\underset{i=1}{\sum }}\left|x_{i}\right|+\overset{n}{\underset{i=1}{\prod }}\left|x_{i}\right|$	30	[-10,10]	0
$f_{3}=\overset{n}{\underset{i=1}{\sum }}{\left(\overset{i}{\underset{j-1}{\sum }}x_{j}\right)}^{2}$	30	[-100,100]	0

**Table 2:** Multimodal function.

Function	Dim	Range	*f*_min_
$f_{4}=\overset{n}{\underset{i=1}{\sum }}\left[x_{i}^{2}-10\cos\left(2\pi x_{i}\right)\right]+10$	30	[-5.12,5.12]	0
$f_{5}=-20\exp\left(-0.2\sqrt{\frac{1}{n}\overset{n}{\underset{i=1}{\sum }}x_{i}^{2}}\right)-\exp\left(\frac{1}{n}\overset{n}{\underset{i=1}{\sum }}\cos\left(2\pi x_{i}\right)\right)+20+e$	30	[-32,32]	0
$f_{6}=\frac{1}{4000}\overset{n}{\underset{i=1}{\sum }}x_{i}^{2}-\overset{n}{\underset{i=1}{\prod }}\cos\left(\frac{x_{i}}{\sqrt{i}}\right)+1$	30	[-600,600]	0

**Table 3:** Comparison of optimization results.

F	IGWO			GWO			PSO		
	Avg	Std	f_min_	Avg	Std	f_min_	Avg	Std	f_min_
F_1_	6.5991E-61	1.0803E-60	9.0538E-64	1.2038E-27	2.154E-27	7.1046E-30	1.62E-04	0.00025071	5.8104E-06
F_2_	1.541E-28	1.3769E-28	8.8133E-30	1.54E-16	9.9257E-17	7.461E-17	4.31E-02	0.02528922	0.00568909
F_3_	2.0747E-46	5.1803E-46	1.0348E-53	6.71E-05	0.00014031	1.0995E-07	8.68E+01	54.2280091	50.162977
F_4_	0	0	0	3.45E+00	3.64620894	5.6843E-14	1.10E+00	0.15524199	0.15523653
F_5_	15.8452336	8.35507149	7.99E-15	9.68E-14	1.35024E-14	7.5495E-14	1.15E+02	136.910361	136.487454
F_6_	0	0	0	2.86E-03	0.00619638	0	9.62E-03	0.0094064	4.2541E-06

**Table 4:** Site selection factor measurements.

	Land price	Rent	Daytime flow	Night flow	High risk area	Number of competitors	Maintenance distance
1	3100	9	9	2	7	1	9
2	2700	7	8	2	7	1	3
3	2500	10	9	2	1	0	2
4	3500	12	2	1	6	2	2
5	2900	12	10	2	5	2	7
6	2900	11	10	2	6	2	2
7	2700	12	10	2	1	1	10

## Data Availability

The labeled data set used to support the findings of this study is available from the corresponding author upon request.
